The article "Aggressive natural killer-cell neoplasm presenting in the marrow: a report of two cases including one with gains of chromosomes 4q and 9p" was published in 2015. Journal: Diagn Pathol.

# Aggressive natural killer-cell neoplasm presenting in the marrow: a report of two cases including one with gains of chromosomes 4q and 9p

**DOI:** 10.1186/s13000-015-0333-x

**Published:** 2015-07-04

**Authors:** Jie-Yang Jhuang, Alexandra Clipson, Yen-Chuan Hsieh, Chun-Chieh Yang, Sheng-Tsung Chang, Ming-Qing Du, Shih-Sung Chuang

**Affiliations:** Department of Anatomic Pathology, Far Eastern Memorial Hospital, New Taipei City, Taiwan; Department of Pathology, University of Cambridge, Cambridge, UK; Department of Pathology, Chi-Mei Medical Centre, 901 Chung-Hwa Road, Yung-Kang District Tainan, Taiwan; Departments of Critical Care Medicine and Pathology, Chi-Mei Medical Center, Tainan, Taiwan; Department of Nursing, National Tainan Institute of Nursing, Tainan, Taiwan; Department of Pathology, College of Medicine, National Taiwan University and Taipei Medical University, Taipei, Taiwan

**Keywords:** Aggressive natural killer-cell leukemia, Bone marrow, Epstein-Barr virus, Extranodal natural killer/T-cell lymphoma, Primary bone marrow lymphoma, T-cell lymphoma

## Abstract

Aggressive nature killer (NK)-cell neoplasm includes aggressive NK-cell leukemia (ANKL) and extranodal NK/T-cell lymphoma (ENKTL), nasal type. ANKL is rare and is characterized by a systemic neoplastic proliferation of NK-cells, usually with a leukemic presentation. ENKTL is a predominantly extranodal lymphoma, occurring mainly in the upper aerodigestive tract. Both are aggressive neoplasms strongly associated with Epstein-Barr virus (EBV). Here we report two patients with aggressive NK-cells neoplasms localized in the bone marrow (BM) who presented as prolonged fever, anemia, and thrombocytopenia. Both were treated initially as infectious disease. Imaging studies revealed splenomegaly without any nodular lesion or lymphadenopathy. BM examination revealed extensive involvement by EBV-positive NK-cells in both cases. Staging workup including nasal examination/biopsy was negative. Both patients passed away in a month. One case showed gains of chromosomes 4q and 9p by array comparative genomic hybridization. Both tumors were diagnostically challenging due to the unusual clinical presentation and absence of leukemic change, tumor mass or lymphadenopathy. Our cases demonstrate that lymphoma should be considered in patients with fever of unknown origin and bone marrow aspiration/biopsy should be performed as early diagnosis and novel therapeutic regimens may benefit these patients.

## Background

In the 2008 WHO classification, aggressive nature killer (NK)-cell neoplasms include 2 entities: aggressive NK-cell leukemia (ANKL) and extranodal NK/T-cell lymphoma, nasal type (ENKTL) [1, 2]. ANKL is rare and characterized by a systemic neoplastic proliferation of NK-cells almost always associated with Epstein-Barr virus (EBV), usually with a leukemic presentation, and an aggressive clinical course. ANKL affects mostly young to middle-aged patients and is more common among Asians. ENKTL is a predominantly extranodal lymphoma occurring mainly in upper aerodigestive tract. It is associated with EBV and has a strong ethnic and geographic predilection, being most common among Asians and Native Americans. The distinction between prototypic ANKL and ENKTL is usually straight forward, yet rare cases with overlapping features may exist. Molecular features have been reported to be different between these entities [3]. Here, we report two cases of aggressive NK-cell neoplasms involving BM but without leukemic phase or extranodal involvement. Furthermore, one case showed gains of chromosomes 4q and 9p by array comparative genomic hybridization (aCGH).

The article "Aggressive natural killer-cell neoplasm presenting in the marrow: a report of two cases including one with gains of chromosomes 4q and 9p" was published in 2015. Journal: Diagn Pathol.

## Case presentation

Case 1 was a 55-year-old Taiwanese female presenting on Oct 18^th^, 2009 with abdominal pain and fluctuating fever for several weeks. There was no prior systemic disease, B symptoms, lymphadenopathy, or skin rashes. Hemograms showed normocytic anemia (hemoglobin at 8.6 g/dL), thrombocytopenia (platelet count at 37,000/μL), and normal white counts without blasts or leukemic cells. Whole body gallium scan revealed increased uptake only at the bilateral lower lung fields but not in the nasopharynx or elsewhere including spleen. Computed tomography (CT) scans of the chest revealed mixed consolidation and ground-glass opacity over bilateral lower lung zones without mass lesions. Empirical antibiotics were administered but in vain. Bone marrow (BM) biopsy was performed on the 9^th^ admission day and ENKTL with extensive marrow involvement was diagnosed. Her serum lactate dehydrogenase (LDH) level was elevated at 395 IU/L (reference: 85–227). Abdominal CT scans were negative for lymphadenopathy or mass lesion in the liver or spleen. Nasal endoscopy and biopsy were negative. Her serum EBV viral load was 130,000 copies/ml. A stage IVB disease with ECOG performance status score of 1 and IPI score of 2 was diagnosed. She received one course of chemotherapy with vincristine and prednisolone but developed metabolic acidosis. Unfortunately, her clinical condition deteriorated rapidly and she died of septic shock with multiple organ failure, five weeks after admission and three weeks after diagnosis.

Table 1 summaries the pathological and immunophenotypic features. By flow cytometry, the marrow lymphocytes expressed CD2, CD56 and cytoplasmic CD3 but not surface CD3, CD5, CD7, CD8 or terminal deoxynucleotidyl transferase, indicating an NK-cell phenotype (Fig. 1a-c). The marrow trephine was hypercellular with a diffuse infiltrate of atypical small to medium-sized lymphocytes accompanied by stromal fibrosis (Fig. 1d and e). Immunohistochemically, the atypical lymphocytes expressed CD3 (Fig. 1f), CD45 and T-cell intracellular antigen (TIA)-1 (Fig. 1g) but not CD2, CD4, CD5, CD7, CD8, CD20, CD30, CD56, βF1, T-cell receptor (TCR)-γ or granzyme B. EBV in situ hybridization (EBER) showed positive signals in around 70 % tumor cells (Fig. 1h). For Infinium genotyping assay, 200 ng DNA isolated from marrow aspirate was hybridized to the HumanCytoSNP-12 Beadchip (Illumina) according to the manufacturer’s instructions. Data were analyzed using the genotyping module of the GenomeStudio software (version 1.9.0; Illumina). Copy-number analysis was performed using the cnvPartition copy-number variation (CNV) analysis plug-in for GenomeStudio software (version 3.2.0; Illumina). A confidence value of greater than 100 was used to determine true copy number changes. The copy number analysis indicated a gain of 1 copy at chromosome 4:83644676 – 4:190742692 (CNV Confidence: 22884.3; Fig. 1i) and a gain of 1 copy in chromosome 9:46587 – 9:21925855 (CNV Confidence: 1630.9) and 9:22098574 – 9:33228189 (CNV Confidence: 2317.0; Fig. 1j) B allele frequency (BAF) plot in both panels demonstrated an altered pattern of BAF (0.0, 0.33, 0.67 and 1.0), while Log R ratio plot displayed no apparent alteration. This was most likely due to the presence of mosaicism in the region of chromosomal gain [4].

The article "Aggressive natural killer-cell neoplasm presenting in the marrow: a report of two cases including one with gains of chromosomes 4q and 9p" was published in 2015. Journal: Diagn Pathol.

**Table 1:** Pathological, immunophenotypical and genotypical findings

	Case 1	Case 2
Cell size	Small to medium	Small to medium
Tumor necrosis	Absent	Present
CD2	-	-
CD3	+	+
sCD3 (FCM)^a^	-	ND
CD4	-	-
CD5	-	-
CD7	-	+
CD8	-	+
CD16	ND	-
CD30	ND	-
CD56	-	-
CD56 (FCM)*	+	ND
TIA-1	+	+
Granzyme B	-	-
βF1	-	-
TCR-γ	-	-
TCR-GR	Polyclonal	Polyclonal

^a^FCM, flow cytometric immunophenotyping using bone marrow aspirate

Abbreviations: ND, not done; sCD3, surface CD3; TCR-GR, T-cell receptor gene rearrangement

**Fig. 1:** Case 1. Flow cytometric analysis of the marrow aspirate shows that the gated atypical lymphocytes express surface CD2 and CD56 but not CD3 or CD7 (**a-c**). In addition, they express cytoplasmic CD3 but not TdT, indicating an NK-cell phenotype. Marrow trephine shows a hypercellular marrow with extensive infiltration by small to medium-sized atypical lymphocytes (**d** and **e**, HE stains; original magnifications × 200 and × 1000, respectively). The tumor cells express cytoplasmic CD3 (**f**), TIA-1 (**g**) and EBER (**h**). Analyses of genomic copy number alteration using the HumanCytoSNP-12 Beadchip (Illumina). **i** and **j**, These two panels show evidence of gain of one copy at 4q21-q35 (**i**) and 9p24-p13 (**j**) respectively. B allele frequency (BAF) plot in both panels demonstrates an altered pattern of BAF (0.0, 0.33, 0.67 and 1.0), which is highlighted in a blue background. Log R ratio plot displays no apparent alteration and this is most likely due to the presence of mosaicism in the region of chromosomal gain

Case 2, a 63-year-old Taiwanese male, presented with abdominal fullness for five days on Sep 25^th^, 2013. Physical examination revealed a flat abdomen devoid of tenderness, rebounding pain or lymphadenopathy. Hemograms showed anemia (hemoglobin at 7.4 g/dL), thrombocytopenia (platelet count at 85,000/μL), and normal white count with presence of myelocytes and nucleated red blood cells (NRBC). There were no blasts or leukemic cells. Laboratory examination revealed elevated LDH level (512 IU/L), abnormal liver and renal function tests, hyperlactatemia, and abnormal inflammatory parameters. CT scans revealed a grade 1 laceration of the slightly enlarged spleen with hemoperitoneum and contrast extravasation without any hepatic lesion or lymphadenopathy. Trans-arterial embolization restored the hemodynamic status with stable hemoglobin level. During hospitalization, lactic acidosis worsened. BM biopsy was performed on the 30^th^ admission day and a diagnosis of ENKTL was made. Serology tests showed elevated EBV-CA IgG, EBV-CA IgA, and EBNA IgG. The serum EBV viral load was 60,000copies/ml. Examination of the upper airway by an otorhinolaryngologist with a nasal biopsy was negative. His ECOG performance status score deteriorated to 4, and he subsequently developed acute oliguric renal failure and hepatic failure. He received only supportive treatment and passed away on the 34^th^ day, one week after pathological diagnosis.

The article "Aggressive natural killer-cell neoplasm presenting in the marrow: a report of two cases including one with gains of chromosomes 4q and 9p" was published in 2015. Journal: Diagn Pathol.

Marrow biopsy of Case 2 showed extensive coagulative necrosis with a remaining small proportion of viable cells at the periphery of the marrow core (Fig. 2a and b). Morphologically, it was difficult to identify the atypical lymphoid cells (Fig. 2c). Immunohistochemical stain with CD3 (Fig. 2d) highlighted the small to medium-sized, polymorphous lymphocytes, including those in the necrotic areas. These cells also expressed CD7, CD8, and TIA-1 (Fig. 2e) and were positive for EBER (Fig. 2f and g) but not CD2, CD4, CD5, CD56, βF1 or TCR-γ. Clonality study for TCR-γ chain gene was polyclonal for both cases using our previously described protocols [5]. There was no fresh/frozen tissue for copy number analysis.

**Fig. 2:** Case 2. Scanning (**a**) and medium-powers (**b**) of the marrow core show extensive coagulative necrosis with scanty viable cells in the right-side end of the core. Even in the high-power view it is difficult to confidently identify the small to medium-sized atypical lymphocytes among the other hematopoietic cells (**c**). The atypical lymphocytes are highlighted by immunohistostaining with CD3 (**d**) with irregular nuclear contours and TIA-1 (**e**). The neoplastic cells are positive for EBV by in situ hybridization (EBER; **f** and **g**, low and high-power views, respectively)

## Discussion

Primary BM lymphoma (PBML) is rare with poorly defined clinicopathological features. Martinez et al. proposed the following criteria for PBML: isolated BM infiltration with no evidence of nodal or extranodal disease and the exclusion of leukemias/lymphomas that are considered to be primarily involving BM [6]. Both of our patients presented as fever of unknown origin (FUO), anemia, and thrombocytopenia and were treated as infectious disease until BM examination. One main question is, if the bone marrow involvement in our cases represent (i) ANKL, (ii) disseminated ENTKL with secondary marrow involvement, or (iii) PMBL. i) ANKL occurs mainly in young adults and shares the same immunophenotype and EBV association with ENKTL. Unlike our cases, patients with ANKL usually have skin rashes, lymphadenopathy, and hepatosplenomegaly and most importantly, leukemic cells in PB [7]. ii) ENKTL with marrow involvement usually occur metachronously or concomitantly with involvement of other anatomical sites such as the aerodigestive tract [8, 9]. In our patients, examination of the upper aerodigestive tract with biopsy was negative. Neither patient had cutaneous or gastrointestinal lesions. Although CT scans revealed splenomegaly in both cases, there was no nodular lesion/mass or lymphadenopathy. Positron emission tomography (PET)-CT is currently the standard for detecting lymphoma but was not performed in our patients [10]. However, both patients received Gallium scan as part of infectious/inflammatory source workup. Although less sensitive, gallium scans were negative in both patients. iii) Accordingly, our cases fit the criteria of PBML of NK-cell origin. Nasal ENKTL may show minimal involvement of the BM and PB at disease dissemination, but extensive marrow involvement is extremely rare [11]. The other differential diagnosis is intravascular lymphoma (IVL), frequently of B-cell phenotype with rare examples of T- and/or NK-cell lineage; and the extremely rare cases with EBV association may share similar immunophenotype with ENKTL [12, 13]. Absence of intravascular pattern in our cases argued against the diagnosis of IVL.

There are only a few reports on genome-wide genetic alterations of aggressive NK-cell neoplasms. Nakashima et al. compared ANKL (n = 10) with ENKTL (n = 17) using array CGH [3]. The recurrent alterations of ANKLs were gain of 1q and loss of 7p15.1-p22.3 and 17p13.1, while that of ENKTL were gain of 2q, and loss of 6q16.1-q27, 11q22.3-q23.3, 5p14.1-p14.3, 5q34-q35.3, 1p36.23-p36.33, 2p16.1-p16.3, 4q12, and 4q31.3-q32.1. They considered ANKL and ENKTL distinct entities based on different genetic alterations. Recently the same group lumped ANKL (n = 9) and ENKTL (n = 27) together and identified two 6q21 regions that were most frequently deleted (14 of 39 or 36 %) using oligo-array CGH and gene-expression profiling [14]. They identified several candidate tumor-suppressor genes that were down-regulated in these regions and their subsequent investigations suggested that two of these suppressor genes, *PRDM1 and FOXO3*, were considered playing an important role in the pathogenesis of NK-cell neoplasms. However, the genetic alterations in our Case one (Chromosomes 4 and 9) were distinct from that in these 2 reports. Studies on more cases are warranted to elucidate the pathogenesis of this rare group of disease.

The article "Aggressive natural killer-cell neoplasm presenting in the marrow: a report of two cases including one with gains of chromosomes 4q and 9p" was published in 2015. Journal: Diagn Pathol.

## Conclusions

In brief, we describe the clinicopathological findings of two aggressive NK-cell neoplasms as PBML with poor outcome, partly due to a delay in diagnosis. Patients with this aggressive neoplasm may benefit from early and accurate diagnosis and administration of novel therapeutic regimens such as SMILE (L-asparaginase, methotrexate, ifosphamide, etoposide, and dexamethasone) protocol, which could overcome the effects of increased P-glycoprotein by the neoplastic NK-cells through the expression of the multi-drug resistance (MDR) gene.

## Consent

The patients have signed consent forms for reporting their diseases.

## Abbreviations

aCGH: Array comparative genomic hybridization
ANKL: Aggressive NK-cell leukemia
BAF: B allele frequency
BM: Bone marrow
CNV: Copy-number variation
CT: Computed tomography
EBER: EBV in situ hybridization
EBV: Epstein-Barr virus
ENKTL: Extranodal NK/T-cell lymphoma
LDH: Lactate dehydrogenase
NK: Natural killer
PBML: Primary bone marrow lymphoma
PET: Positron emission tomography
TCR: T-cell receptor
